# Overexpression of the Insulin Receptor Isoform A Promotes Endometrial Carcinoma Cell Growth

**DOI:** 10.1371/journal.pone.0069001

**Published:** 2013-08-07

**Authors:** Chun-Fang Wang, Guo Zhang, Li-Jun Zhao, Wen-Juan Qi, Xiao-Ping Li, Jian-Liu Wang, Li-Hui Wei

**Affiliations:** Department of Obstetrics and Gynecology, Peking University People’s Hospital, Peking University, Beijing, China; Clermont Université, France

## Abstract

Epidemiological studies have demonstrated that type 2 diabetes mellitus (T2DM) and hyperinsulinemia are associated closely with endometrial carcinoma risk, although the molecular mechanism remains unclear. Insulin receptor isoformA expression is upregulated in many cancer cells and tissues, which suggests that IR-A-mediated signaling pathways may have important implications for cancer pathogenesis. We measured the expression of insulin receptor isoforms (IR-A and IR–B in the normal endometrium tissues, the endometrial carcinoma tissues and the endometrial carcinoma cell lines. We found that the total insulin receptor (IR) and IR-A expression mRNA levels and the ratio of IR-A to total IR in endometrial carcinoma specimens were significantly higher than them in control endometrial tissue specimens(P<0.05). Further analysis indicated that the tendency was more prominently in patients with T2DM. IR-A mRNA was differentially expressed in four endometrial carcinoma cell lines (Ishikawa, KLE, RL95-2 and HEC-1-A. RL95-2 cells have a low endogenous IR-A expression, and these were used to construct a stable cell line overexpressing IR-A. We found that IR-A overexpression significantly increased cell proliferation, the proportion of cells in S phase, activation of the Akt pathway and tumorigenicity of xenografts in nude mice. In contrast, there was no significant difference in the the percentage of apoptotic cells between cells overexpressing IR-A and control cells. Moreover, levels of phosphorylated ERK1/2 protein were significantly decreased in cells overexpressing IR-A relative to controls. These findings reveal the pivotal role of IR-A in endometrial cancer carcinogenesis, and suggest that the association of elevated IR-A levels with cell proliferation and tumorigenicity may be causally linked to its effect on the proportion of cells in S phase and the activation of the Akt pathway.

## Introduction

Endometrial cancer is the third most common malignancy of the female genital tract reported in China. The incidence and mortality rate of endometrial carcinoma has increased in recent years [1]. An improved understanding of the factors regulating endometrial cancer cell growth should lead to better treatment options.

The insulin receptor (IR) belongs to a subfamily of receptor tyrosine kinases that includes the insulin-like growth factor (IGF) 1receptor(IGF-1R) and the insulin-receptor-related receptor. Members of this family of receptors are tetrameric proteins consisting of two extracellular α-subunits and two transmembrane β-subunits linked by disulfide bonds [2]. The human IR is encoded by a large single insulin receptor gene comprising 22 exons and the protein is expressed as two different isoforms that differ at the carboxyl terminus of the α-subunits by 12 amino acids [3]. The presence (IR–B, or IR exon 11+) or absence (IR-A, or exon 11-) of these residues alters the functional properties of the isoform. IR–B is a classical IR that regulates glucose uptake. In contrast, IR-A has potent mitogenic and anti-apoptotic functions and plays a key role in cell proliferation [4].

Expression of the insulin receptor isoform A (IR-A) has been predominantly detected in cancers of the breast, lung, colon [5], thyroid [6], ovaries [7], and smooth and striated muscle [8]. IR-A expression is upregulated in many cancer cells and tissues, which suggests that IR-A-mediated signaling pathways may have important implications for cancer pathogenesis [9]. Understanding the IR-A expression and function in the endometrial cancer tissues and cells is critical for advancing our knowledge of endometrial cancer biology, and could lead to the development of novel tumor-specific therapies.

The present study aims to determine the expression of IR-A in the normal endometrium tissues, the endometrial carcinoma tissues and the cell lines. endometrial carcinoma tissues, and endometrial carcinoma cell lines (Ishikawa, KLE, HEC-1-A and RL95-2, which was named RL95-2-CON in this paper). Thenwe explored the role of IR-A in human endometrial cancer development.

## Results

### Expression of insulin receptor isoforms and IGF-2 in endometrial cancer cell lines and tissues

To assess expression of IR and IGF-2 in human endometrial cancer cell lines, reverse transcription polymerase chain reaction (RT-PCR) and Real time RT-PCR were performed using RNA from the HEC-1-A, Ishikawa, KLE, RL95-2-CON endometrial cancer cell lines, positive control Liver cancer cell line Hep-G2 and breast cancer cell line MCF-7. RT-PCR shown that IR-A, IR–B and IGF-2 are differentially expressed in HEC-1-A, Ishikawa, KLE and RL95-2-CON endometrial cancer cells(Figure 1A). The real time RT-PCR results shown the relative expression levels of IR-A and total IR in four endometrial cancer cells (Figure 1B). The ratio of IR-A to total IR which got from the real time RT-PCR results was highest in Ishikawa cells and reduced in HEC-1-A, KLE and RL95-2-CON cells(Figure 1C).

**Figure 1:** IR-A expression in endometrial carcinoma cell lines. A. Expression of IR-A (444 bp), IR–B (480 bp), IGF-2 (214 bp) and GAPDH (226 bp) mRNA in endometrial carcinoma cell lines was measured by RT-PCR. The results indicates that two transcript isoforms of insulin receptors (IR-A and IR–B) and IGF-2 were co-expressed in HEC-1-A, Ishikawa, KLE and RL95-2–CON cells. RL95-2–CON has a much higher ratio of IR–B expressed than IR-A. B. Real-time RT-PCR indicates the relative levels of IR-A and total IR mRNA in endometrial carcinoma cell lines, normalized to GAPDH. C.The ratio of IR-A/ IR in endometrial cancer cell lines from real-time RT-PCR results. D. ELISA quantitation of IGF-2 protein secreted by RL95-2–CON, RL95-2–IR-A, KLE, HEC-1-A and Ishikawa cells.

Previous studies have reported that IR-A is a high affinity receptor for IGF-2 [10], To further confirm whether the endometrial cancer cell lines can secrete IGF-2, enzyme-linked immunosorbent assay (ELISA) was performed using cell culture supernatants from the HEC-1-A, Ishikawa, KLE, RL95-2-con and RL95-2-IR-A cell lines. We observed that IGF-2 secretion was highest in RL95-2–CON cells and reduced in RL95-2–IR-A, KLE, HEC-1-A and Ishikawa cells. There was no difference in IGF-2 secretion between RL95-2–CON and RL95-2–IR-A cells(Figure 1D).

RT-PCR results of tissue specimens shown that mRNA encoding IR-A was expressed in 78 of the 103 endometrial carcinoma samples(75.7%) and in 21 of the 60 normal endometrial tissue samples(35%) and the electrophoretic assay of representative examples was shown in Figure 2.

**Figure 2:** Expression of IR-A/ IR–B in endometrial carcinoma tissues and control normal endometrium tissues. A. Representative examples of the endometrial carcinoma tissues (total 103cases). Lane M shown the DNA marker and Lanes T1–T19 correspond to 19 separate endometrial carcinoma patients B. Representative examples of control normal endometrium tissues(total 60 cases). Lanes N1–N25 correspond to 25 separate patients with normal endometrium.

Real time RT-PCR results of tissue specimens was shown in table 1, The total IR and IR-A expression levels and the ratio of IR-A to total IR in endometrial carcinoma specimens were significantly higher than them in control endometrial tissue specimens(P<0.05). Further analysis indicated that the tendency was more prominently in patients with type 2 diabetes mellitus (T2DM) (table 2).

**Table 1:** Relative expression levels of IR and IR-A in endometrial cancer and control endometrial tissues.

	**IR / GAPDH**	**IR-A / GAPDH**	**IR-A / IR**
endometrial cancer	0.018821±0.013805	0.012744±0.011868	0.62964±0.196977
Control endometrial tissues	0.013779±0.012518	0.00827±0.009825	0.502148±0.17704
*P* value	<0.05	<0.05	<0.05

**Table 2:** Relative expression levels of IR and IR-A in endometrial cancer and control endometrial tissues from patients with type 2 diabetes mellitus.

	**IR / GAPDH**	**IR-A / GAPDH**	**IR-A / IR**
endometrial cancer	0.02224±0.011295	0.014868±0.007912	0.68192±0.193396
Control endometrial tissues	0.016076±0.014604	0.009154±0.012137	0.5391±0.18775
*P* value	<0.05	<0.01	<0.01

### Overexpression of IR-A in RL95-2-CON cells

To investigate the role of IR-A in endometrial carcinogenesis and the potential interaction with T2DM signalling pathway, we synthesized stable RL95-2-CON cells that overexpressed IR-A because IR-A mRNA expression in the parental RL95-2-CON cell line is low. Full-length IR-A cDNA was cloned into the pcDNA3.1 eukaryotic expression plasmid (IR-A–pcDNA3.1) and used to construct the RL95-2-CON cell line stably overexpressing IR-A (RL95-2–IR-A).

The IR-A mRNA expression in one cloning of the RL95-2–IR-A stable cell line was determined to be 111.41 times higher than in parental cells by real-time RT-PCR and this cloning was used in the follow-up experiments.

### IR-A overexpression enhances cell proliferation

To investigate the effect of IR-A overexpression on cell proliferation, we plotted 7-day growth curves for RL95-2–IR-A, RL95-2–CON and RL95-2–NC using OD490 nm values, The growth curves for RL95-2–CON and RL95-2–NC were similar, but IR-A overexpression significantly enhanced the proliferation of RL95-2-CON cells when plated 2000 cells/well starting cells(Figure 3A). According to OD490 nm values at 72 hours when plated different number of starting cells, we observed that IR-A overexpression can’t significantly enhanced the proliferation of RL95-2-CON cells when plated 10000 cells/well or more starting cells(Figure 3B).

**Figure 3:** IR-A overexpression increases cell proliferation rate. A. Proliferation of RL95-2–IR-A, RL95-2–CON and RL95-2–NC cells was measured over a 7-day period (plate 2000 cells/well as starting cells) B. Proliferation of the three cells was measured after 72 hours (plate 2000, 5000, 10000, 20000 cells/well as starting cells). 6 replicate wells were included per sample and the data points were present as means±SD. *, *P* < 0.05 vs. control.

### IR-A overexpression leads to increased cell division

To determine whether the IR-A overexpression could influence the cell cycle progression of RL95-2-CON cells, flow cytometry was used to quantitate the proportion of RL95-2–IR-A cells containing in S phase DNA content relative to controls. We found that 25.65% and 26.39% of RL95-2–CON and RL95-2–NC cells, respectively, were in contained S phase cells, but that this was increased to 35.04% in RL95-2–IR-A cells (Figure 4A, C). The proportion of RL95-2–IR-A cells containing S phase DNA content was significantly higher than controls (*P*<0.05).

**Figure 4:** IR-A overexpression affects cell cycle parameters. A. Flow cytometry analysis of the S phase DNA content in RL95-2-IR-A, RL95-2–CON and RL95-2–NC samples. B The percentage of apoptotic cells in three cells. C,D. The proportion of cells containing S phase DNA and the percentage of apoptotic cells are presented as means±SD. *, *P* < 0.05 vs. control.

To further investigate the potential anti-apoptotic role of IR-A in endometrial carcinoma, we used a double labeling technique using Annexin-V and PI to distinguish between apoptotic and necrotic cells. The percentage of apoptotic cells was 5.47% and 5.32% in the RL95-2–CON and RL95-2–NC control cells, but was reduced to 4.59% in RL95-2–IR-A cells (Figure 4B, D). There was no significant difference of the percentage of apoptotic cells between RL95-2–IR-A and control cells(*P*>0.05).

### PI3K-Akt and ERK signaling are differentially regulated in cells overexpressing IR-A

As no IR-A specific antibodies are available, we conﬁrmed that expression of IR-A protein was increased in RL95-2–IR-A cells by quantitating the total insulin receptor expression using an insulin receptor (IR) pan-specific antibody. As shown in Figure 5A, B. IR protein expression in RL95-2–IR-A cells was approximately three-fold higher than in either RL95-2–CON or RL95-2–NC cells.

**Figure 5:** Effect of IR-A overexpression on downstream signaling pathways. A. Western blot analysis of IR protein expression and expression of downstream signaling proteins in RL95-2-CON, RL95-2–NC and RL95-2–IR-A cells. B. IR protein expression in RL95-2–IR-A cells is significantly higher than that in RL95-2–CON and RL95-2–NC cells. C. The relative expression of phospho-Akt is signiﬁcantly increased and the relative expression of phosphorylated ERK1/2 reduced in RL95-2–IR-A cells than controls. *, #, *P* < 0.05 vs. control.

The PI3K-Akt and ERK signaling plays a role in the regulation of various cellular processes such as proliferation, differentiation, development, survival and apoptosis [11]. So we measured phospho-ERK1/2, phospho-Akt and total ERK1/2 and Akt to detect the activation of these two signaling pathways. Total ERK1/2 and Akt protein expression were not affected by IR-A overexpression. However, levels of phospho-Akt were signiﬁcantly increased in RL95-2–IR-A cells relative to controls, while levels of phospho-ERK1/2 were reduced (Figure 5C).

### Inhibition of the PI3K–Akt pathway reverses the effects of IR-A overexpression

In order to confirm the results that IR-A -induced cell proliferation through PI3K/Akt pathway, we treat the RL95-2–IR-A cells with PI3K inhibitor (LY294002) [12].

Levels of phosphorylated Akt were reduced 48 h after treatment with 5, 10, 20 or 40 µM LY294002. Further, the proportion of RL95-2–IR-A cells in S phase was reduced and the proliferation rate of RL95-2–IR-A cells was reduced 48 h after treatment with 20 µM LY294002(Figure 6).

**Figure 6:** PI3K inhibition reverses the effects of IR-A overexpression. A. Western blot analysis of phospho-Akt and total Akt levels 48 h after treatment with 5, 10, 20 and 40 µM of LY294002. B. Growth curves of RL95-2–IR-A cells following treatment with 20 µM LY294002 and without. C. Flow cytometry analysis indicating the proportion of RL95-2–IR-A cells containing S phase DNA at 48 h after treatment with 20 µM LY294002. D. Flow cytometry analysis indicating the percentage of apoptotic cells in RL95-2–IR-A cells at 48 h after treatment with 20 µM LY294002. *, *P* < 0.05 vs. control.

### IR-A overexpression increases tumorigenicity of endometrial carcinoma cells

To explore whether IR-A overexpression in RL95-2-CON cells affects their tumorigenicity of nude mice xenografts, we injected RL95-2-IR-A, RL95-2–CON or RL95-2–NC cells into BALB/c nude mice and monitored tumor volumes every week for 5 weeks. As shown in Figure 7, there are subcutaneous tumor in all three group mice and the histology of tumours was endometrial carcinoma. RL95-2–IR-A xenografts developed larger tumors than those of RL95-2–CON and RL95-2–NC control cells, indicating that 1R-A overexpression exerts a strong tumor-promoting effect on endometrial carcinoma cells in vivo.

**Figure 7:** Tumorigenicity of the RL95-2–IR-A, RL95-2–CON and RL95-2–NC cells in a xenograft model. A. Photographs of the inoculated BALB/c nude mice five weeks after inoculation, showing the tumor size. B. RL95-2–IR-A, RL95-2–CON and RL95-2–NC cells were injected groups of five mice and tumor volumes were measured using calipers every week after the inoculation. C. Five weeks after inoculation, tumors were excised, fixed, and stained by hematoxylin and eosin (H&E; 400× magnification). *, *P* < 0.05 vs. control.

## Discussion

In this study, we investigated the role of IR-A in endometrial carcinogenesis in vitro and in vivo. We found that IR-A is expressed at similar levels in normal endometrial tissues, endometrial carcinoma tissues and endometrial carcinoma cells. However, further analysis showed that IR-A expression was significantly higher in endometrial carcinomas from patients with T2DM than that in control patients. A number of epidemiological studies have demonstrated that type 2 diabetes mellitus (T2DM) is an important risk factor for many cancers, including endometrial carcinoma, although the molecular mechanism remains unclear [13]. the insulin receptor (IR) have been found to be overexpressed in cancer cells [14,15] and signaling through IR is increased in hyperinsulinemia [16]. Several studies have firmly established that IGF-2 elicits its biological effects through IR-A. For instance, IGF-2 is a more potent mitogen than insulin in mouse fibroblasts expressing only IR-A and not IGF-IR (R-/IR-A cells) [4].

Previous studies have also shown that endometrial carcinomas can express IGF-2 [17]. Interestingly, we confirmed that endometrial carcinoma cells, and particularly the RL95-2-CON cell line, secrete IGF-2 by RT-PCR and Elisa. Taken together, these data support that IR-A overexpression drives endometrial carcinogenesis, and we additionally propose that increased IGF-2 secretion in cells overexpressing IR-A may further stimulate the IR pathway.

Our study also shown that cell lines with overexpression of IR-A(RL95-2-IR-A) was successfully constructed and overexpression of IR-A showed a significant proliferation-promoting effect in vitro on RL95-2-CON cell lines which originally has a low expression level of IR-A. Flow cytometry analysis shown that one possible cause of cell growth faster in RL95-2–IR-A may be due to the DNA content in S phase increased. The xenotransplant nude mice model datas shown that the average tumor volume in RL95-2–IR-A xenotransplant mice group were signiﬁcantly bigger than those in the control group indicating that the IR-A could increased the growth of RL95-2-CON cells in vivo. We discovered that the PI3K/Akt signaling pathway was activated and and the MAP kinase pathway was inactivated in cells overexpressing IR-A level, indicating that IR-A-mediated proliferation occurs through the PI3K/Akt signaling pathway and not the MAP kinase pathway. The PI3K/AKT axis regulates essential cellular functions including cell survival, proliferation, migration, and angiogenesis [18]. the PI3K-Akt signaling pathway is implicated in human diseases including diabetes and cancer. Dysregulation and activation of the pathway is common in a large fraction of most human tumor types [19]. Further, PI3K-Akt pathway inhibition led to a reduction in Akt phosphorylation, a reduction in the proportion of cells in S phase and a reduction in growth rate of cells overexpressing IR-A. Our hypothesis may be perfect for that IR-A overexpression drives endometrial carcinogenesis through the PI3K/Akt signaling pathway.

In conlusion, IR-A expression in endometrial carcinoma patients with T2DM was significantly higher than that in patients without T2DM, and it is likely that IR-A overexpression can promote endometrial carcinoma cell proliferation. It is possible that the level of IR-A expression could make a significant contribution to cell growth and survival in endometrial carcinomas. However, the speciﬁc pathogenesis and molecular mechanism requires further investigation.

## Materials and Methods

### Reagents

CellTiter 96® AQueous One Solution Cell Proliferation Assay was purchased from Promega (USA). The Annexin V-FITC & PI Apoptosis Detection Kit was purchased from Beijing Puli Lai Gene Technology Co. Ltd (China). The anti-insulin receptor antibody was purchased from Abcam (Cambridge, UK); anti-phospho-p44/42 MAP Kinase (Thr202/Tyr204), anti-p44/42 MAPK, anti-phospho-Akt (Ser473), anti-Akt, anti β-actin and anti-rabbit IgG horseradish peroxidase (HRP)- conjugated antibodies were purchased from Cell Signaling Technology (Beverly, MA, USA). LY294002 was purchased from Invitrogen (Carlsbad, CA, USA).

### Tissue samples and cell lines

With approval from the ethics committee for research involving Human Subjects of Peking University People’s Hospital and patients’ written informed consent, Samples of 103 endometrial carcinomas were obtained from patients treated with surgery in the Peking University People’s Hospital from November 2007 to July 2011. 18 of them are patients with type 2 diabetes mellitus (T2DM). 60 normal endometrial tissues were obtained from patients who received hysterectomy for early stage ovarian cancer or early stage Cervical Cancer during the same period. 9 of them are patients with T2DM. The tissue samples were immediately snap frozen and stored at liquid nitrogen. All endometrial carcinomas and normal endometrial tissues were review confirmed by two pathologists. The mean ages of patients with endometrial carcinomas and controls were 61 ± 11 years and 56± 14 separately. The difference was not statistically significant.

Ishikawa, HEC-1a, KLE and RL95-2-CON endometrial cancer cell lines were obtained from the American Type Culture Collection (Manassas, VA, USA) and maintained in our laboratory. Breast cancer cell line MCF-7 was donated by Professor Mao Zebin in department of Biochemistry, Peking University Basic Medical School and Liver cancer cell line Hep-G2 was donated by Hepatobiliary Surgery Center of Peking University People’s Hospital, both of them was obtained from American Type Culture Collection initially. All cell lines were maintained under 5% CO_2_ at 37° C in appropriate culture medium containing 10% fetal bovine serum (FBS) (Hyclone, Logan, UT). Ishikawa, HEC-1a, MCF-7, and Hep-G2 cells were cultured in DMEM and KLE and RL95-2-CON cells were cultured in DMEM/F12 (Gibco-BRL, Gaithersburg, MD).

### Reverse transcription polymerase chain reaction (RT-PCR) and real-time RT-PCR

Total RNA was prepared from endometrial cancer cells and frozen tissue samples using Trizol reagent (Invitrogen, USA) and cDNA was synthesized from 2 µg total RNA using a QuantScript RT Kit (Tiangen, China), and used for PCR ampliﬁcation. Two pairs of primers were used to amplify the insulin receptor isoforms. F1,5’-AGG CAG GCG GAA GAC AGT-3’ and R1,5’-GAT GCG ATA GCC CGT GAA-3’ ampliﬁed IR-A and IR–B mRNA fragments of 444 bp and 480 bp, respectively; F2,5’-AAC CAG AGT GAG TAT GAG GAT-3’ and R2,5’-CCG TTC CAG AGC GAA GTG CTT-3’ ampliﬁed IR-A and IR–B mRNA fragments of 600 bp and 636 bp, respectively. Primers used to amplify IGF-2 were F,5’-CTG TGC TAC CCC CGC CAA GT-3’ and R,5ʹ-ACG TTT GGC CTC CCT GAA CG-3’, producing a 214 bp fragment. As a control, glyceraldehyde 3-phosphate dehydrogenase (GAPDH) was ampliﬁed using the primers F,5’-GAA GGT GAA GGT CGG AGT C-3’ and R,5’-GAAGATGGTGATGGGATTTC-3’, producing a 226 bp fragment.

To accurately quantify insulin receptor mRNA expression, IR-A, IR and GAPDH cDNAs were ampliﬁed using real-time PCR. Primers, probe and PCR Master Mix (GAPDH, IR-A, IR) were purchased from Applied Biosystems (USA). All reagents were kept on ice and the probe mix was kept in the dark. PCR conditions were: 50° C for 2 min, 95° C for 10 min, then 40 cycles of 92° C for 15 s and 60° C for 60 s. The comparative Ct method was used to calculate the relative differences in mRNA expression.

### Enzyme-linked immunosorbent assay

IGF-2 protein secretion was measured in culture medium using a commercially available enzyme-linked immunosorbent assay (ELISA) kit (R and D Systems). The detection limit of the kit is 15 pg/mL.

### Construction of RL95-2-CON cell lines overexpressing IR-A

Full-length IR-A cDNA was amplified from the INSR-TOPO-XL (BC117172) plasmid using high-fidelity DNA polymerase, cloned into the pcDNA3.1 eukaryotic expression vector (Invitrogen, USA) and verified by restriction digest (two bands of the expected sizes, 5.5 kb and 4 kb) and sequencing. The IR-A–pcDNA3.1 plasmid was transformed into *E. coli* MAX DH10B and amplified, then transfected into RL95-2-CON cells using Lipofectamine 2000 (Invitrogen, USA). Stably transfected cell clone were done using G418 scanning. Western blot and RT PCR analysis for detecting IR-A protein and mRNA in stably transfected cell clone.

Stable cells clone containing IR-A–pcDNA3.1 were named RL95-2–IR-A; those containing empty pcDNA3.1 plasmid were named RL95-2–NC; and the parental cell line was named RL95-2-CON.

### Cell proliferation

The MTS assay was used to generate 7-day growth curves and OD 490nm at 96h for RL95-2–CON, RL95-2–NC and RL95-2–IR-A cell lines, according to the protocol for the CellTiter 96® AQueous One Solution Cell Proliferation Assay. The proliferation rate of RL95-2–IR-A cells treated with 0 or 20 µM of the PI3K inhibitor LY294002 for 48 h was also established. Each treatment was administered to cells at the same time in six individual wells per experiment, and the experiments were repeated three times.

### Flow cytometry

Cells (5 x 10^5^) were seeded into 6-well plates and incubated overnight in DMEM/F12 containing 10% FBS, and then harvested for flow cytometry analysis as described previously [20]. Chilled ethanol (4° C) was added to the cell suspension to a final concentration of 70% and incubated at 4° C overnight. After washing, cells were resuspended in PBS and strained through a 400-µm mesh sieve (Wako, Osaka, Japan) to exclude cell aggregates. RNase (100 µg/ml final concentration) was added to the cell suspension and incubated at 37° C for 30 min in the dark. Cells were then stained with propidium iodide (PI; 100 µg/ml) in PBS for 30 min at room temperature. The DNA content of cell samples was measured using a FACSCalibur flow cytometer (Becton Dickinson, Mountain View, CA, USA). Apoptotic cells were detected according to the flow cytometry protocol of the Annexin V-FITC & PI Apoptosis Detection Kit (Beijing Biosea Biotechnology Co., Ltd, China) using a FACSCalibur flow cytometer.

Cell cycle progression was determined for RL95-2–IR-A cells treated with 0 or 20 µM of LY294002 for 48 h.

### Western blot analysis

RL95-2–IR-A,RL95-2–NC and RL95-2–CON cells were harvested and protein extraction was performed as described previously [21]. Protein concentration was determined using a BCA Protein Assay Kit (Pierce Biotechnology, Rockford, IL, USA) according to the manufacturer’s instructions. Soluble protein (30 µg) was separated on a 10% SDS-PAGE gel, and then transferred to a polyvinylidene difluoride (PVDF) membrane (Millipore, USA). Membranes were blocked by incubation with 5% skimmed milk in Tris-buffered saline containing 0.1% (v/v) Tween-20 (Sigma-Aldrich, St. Louis, MO, USA; TBS-T) at room temperature for 2 h. Phosphorylated ERK1/2, total ERK1/2, phosphorylated Akt, total Akt and β-actin proteins were detected by incubating membranes overnight at 4^°^ C with the relevant antibodies (1:1000 dilution) in TBS-T containing 5% BSA. After washing three times for 5 min with TBS-T, membranes were incubated for 2 h at room temperature with HRP-conjugated secondary antibody (1:5000 dilution) in TBS-T containing 5% skimmed milk. Proteins were detected using the ECL Plus Western blotting detection system (GE Healthcare, Chalfont St. Giles, UK). Protein band intensity was measured using the MicroChemi chemiluminescence gel imaging system (Israel DNR).

RL95-2–IR-A were treated with 0, 5, 10, 20 or 40 µM LY294002 PI-3K inhibitor for 48 h, then phospho-Akt expression was measured by Western blotting

### Xenograft assay

In vivo studies were performed in athymic nude mice to examine the tumorigenicity of control RL95-2-CON and IR-A-overexpressing cells. Female four-week-old BALB/c nude mice were obtained from the Beijing Vital River Laboratory Animal Technology Co Ltd (Certificate No: SCXK 2006-0008) and maintained in speciﬁc pathogen-free facilities approved by the Animal Care and Use Committee of Peking University People’s Hospital. Nude mice were randomly divided into three groups (five mice per group). RL95-2-IR-A, RL95-2-NC or RL95-2-CON cells (5×10^6^) were inoculated subcutaneously into the right ﬂank of each mouse. Tumor growth was measured weekly using vernier calipers and tumor volume was calculated using the formula [4]: length (mm) × width^2^ (mm^2^)/2. Animals were sacriﬁced five weeks post- inoculation. Tissue samples were harvested for histological analysis, ﬁxed and embedded in parafﬁn wax, and 3 µm sections were cut.

### Statistical analysis

All statistical analyses were performed using SPSS13.0 software (SPSS, Chicago, IL, USA). Comparisons among all cell groups were performed using one-way analysis of variance (ANOVA) and P-Values less than 0.05 was considered to be statistically signiﬁcant. The Tukey’ post hoc test was used for samples where differences were statistically signiﬁcant.
